This article has been retracted.

# Impact of the third wave of the COVID-19 pandemic and interventions to contain the virus on society and patients with kidney disease in Cambodia

**DOI:** 10.1186/s41100-021-00372-6

**Published:** 2021-10-09

**Authors:** Tam Nov, Toru Hyodo, Yukie Kitajima, Kenichi Kokubo, Toshihide Naganuma, Haruki Wakai, Akihiro Yamashita, Elin Phon, Hideki Kawanishi

**Affiliations:** 1 International University (IU), Phnom Penh, Cambodia; 2 Cambodia Association of Nephrology (CAN), Phnom Penh, Cambodia; 3 NGO Ubiquitous Blood Purification International (NGO UBPI), Yokohama, Japan; 4 Japanese Assistance Council for Establishing Dialysis Specialists’ System in Cambodia, Yokohama, Japan; 5 Department of Urology, Osaka City University, Osaka, Japan

**Keywords:** SARS-CoV-2, COVID-19, Lockdown, Cambodia, Hemodialysis patients, End-stage renal disease, Chronic kidney disease, Food insecurity, COVID-19 vaccination, Socioeconomic hardship, Health workers in nephrology

## Abstract

Cambodia detected its first case of COVID-19 just 3 days before WHO declared that the outbreak constituted as PHEIC. As of February 15, 2021, and after two major outbreaks, only 479 cases had been reported, 396 (83%) of which were imported. This small number of cases was largely thanks to stringent measures and policies put in place by the government to curb the spread. Despite these efforts, a third cluster outbreak was declared on February 20, 2021. It has disrupted all aspects of life in Cambodia. As in many other countries affected by the virus, economic hardship, lockdowns in cities, and food insecurity ensued. Against the backdrop of this widespread impact on the citizens of Cambodia, we conducted this review article to better understand the situation of healthcare workers in nephrology and dialysis patients and the challenge they face in providing and receiving essential medical care. Healthcare providers have continued working to serve their patients despite facing a high risk of catching SARS-CoV-2 and other challenges including difficulties in traveling to work, increased physical and mental burden, and higher stress due to measures taken to minimize the risk of transmission during patients’ care. Some healthcare workers have been discriminated against by neighbors. The most difficult mission is when having to deal with families whose loved one is denied access to a hemodialysis session due to suspected COVID-19 while waiting for PCR test results. Hemodialysis patients reported facing economic hardship and increasingly difficult circumstances. When access to food is limited, patients have eaten canned or dried salted food rather than an appropriate hemodialysis diet. Because hemodialysis centers are concentrated in a few cities, access has become even harder during the travel ban. In-center hemodialysis rules are stricter and does not allow family members or escorts to enter the unit. Only a few hemodialysis patients have been vaccinated. Before COVID-19, hemodialysis patients already faced major burdens. The pandemic appears to be decreasing their quality of life and survival even further. Through this study, we have revealed current hardships and the need to improve the situations for both healthcare workers in nephrology and hemodialysis patients in Cambodia.

## ESKD and hemodialysis in Cambodia before COVID-19

In 2017, there were an estimated 7 hemodialysis centers, both public and private, in Cambodia [1]. The number has been growing, but the exact amounts and locations of those centers have been reported more recently. The centers are thought to be concentrated in Phnom Penh, Battambang, Siem Reap, and Kampong Cham Province (Fig. 1), out of 25 cities and provinces nationwide [1, 2]. To receive treatment, patients from provinces have to travel to Phnom Penh for each treatment session, and costs are generally paid out-of-pocket by most patients, as there is no national insurance system to cover hemodialysis [1, 3].

**Fig. 1:** Map shows current locations of hemodialysis centers within Cambodia. Adapted from Ref. [30]

## General information about COVID-19 in Cambodia

Cambodia detected its first case of COVID-19 on January 27, 2020 [4], just 3 days before the World Health Organization declared that the outbreak constituted a Public Health Emergency of International Concern (PHEIC) [5, 6]. Despite having a weak healthcare system compared with other countries in Southeast Asia and being a resource-limited country, Cambodia is among the countries with the lowest number of COVID-19 cases in 2020 (Fig. 2) and early 2021 [7].

**Fig. 2:** Graph shows number of cases in 2020. Cases spike in March and November 2020. Adapted from Ref. [28]

Since early in the pandemic, the Royal Government of Cambodia has put in place many measures and policies to stop the spread of the virus. The country isolated itself from the rest of the world by requiring all incoming travelers to have negative COVID-19 health certificates, carry medical insurance, undergo PCR testing on arrival, stay in quarantine for 14 days, and undergo further testing on day 13. Although internal movement and economic activities within the country were not restricted, the public was encouraged to adopt public health measures like mask wearing, frequent handwashing, and social distancing [8]. For a long time, these measures were effective. As of February 15, 2021, 396 (83%) of the 479 reported cases were imported and the remaining cases were locally acquired. No clusters of undiagnosed respiratory illness were reported to a national hotline, and influenza-like illnesses and severe respiratory illness reports were below expected levels in February 2021 [9].

A new cluster outbreak was declared by the government on February 20, 2021, marking the third outbreak of community transmission in Cambodia [10, 11]. Since then, all aspects of life in the country have been impacted by the course of this outbreak (Fig. 3). As in many other countries affected by the virus, economic hardship, lockdown in cities, and food insecurity ensued [12, 13]. As of the time of writing (May 15, 2021), there have been a total of 22,184 cases and 150 deaths, and these numbers are expected to rise further [10, 14]. In response, the government has attempted to accelerate its vaccination campaign, especially for residents in hotspot areas. To date, 2.13 million adults have been vaccinated, or about 21% of the target population [14]. According to National Deployment and Vaccination Plan for COVID-19 vaccines, there are 8 target groups with different priorities to receive the vaccine [15]. Unfortunately, ESKD patients and patients with hemodialysis vaccination information could not be found in this important document.

**Fig. 3:** Number of COVID-19 cases in early 2021. New cluster outbreak declared on February 20, 2021. Adapted from Ref. [7]

Because of the slowdown of the global economy, factories around the world have shut down, disrupting supply and demand chains. Cambodia's economy saw the economy contract by − 3.1% in 2020, a number the country has not seen for more than 20 years [6, 16, 17]. It is estimated that 135,000 garment workers and 17,000 tourism workers lost their job due to the impact of the pandemic, but the true number could be higher. The situation is even worse for workers in the informal sector such as street vendors, hairdressers, and tuk tuk and motorbike taxi drivers [6, 12].

To slow the spread of the virus, The Royal Government of Cambodia has imposed a lockdown in high-risk areas (Fig. 4), banned interprovincial travel, restricted internal movement within areas, and restricted international travelers, as governments around the world have done [12, 18]. Despite the good intentions of these measures, they have resulted in collateral damage to citizens, especially those in disadvantaged communities and rural areas [6, 9, 12].

**Fig. 4:** Map shows high-risk area under strict lockdown in Phnom Penh. There were 3 designated zones effective from April 29 to May 5, “yellow, orange, and red,” and each has limited different travel capability. Red zone means no one is allowed to get out of the house. Adapted from Ref. [29]

## The overview of COVID-19 effects on society

A few hours before lockdown was announced in the capital Phnom Penh and Takhmao City, people flocked to the markets to buy as much food as they could afford (Fig. 5) because of food insecurity [12, 19]. In the areas with the most restrictive lockdown measures, called “red zones”, residents experienced food shortages and took to the streets in protests (Fig. 6) [13, 20]. Fruits and vegetables were in short supply, as were medical supplies and daily necessities. Suppliers could not bring products to the affected areas and people could not easily leave home, main public markets all closed and the prices of products soared. Thus, residents could not readily meet their basic needs [21].

**Fig. 5:** People flock to markets in Phnom before the lockdown (April 14, 2021)

**Fig. 6:** Protests in a “red zone” (May 13, 2021). Citizens in a “red zone” who had difficulty accessing food and supplies take to the streets to protest

The pandemic created a dramatic surge in demand for masks, alcohol, personal protective equipment (PPE), and other medical supplies. However, as most of these supplies are imported, the prices have been extremely high, far beyond what most Cambodians could afford [21, 22]. Counterfeit medical supplies have also been a problem, such as hand sanitizer made with methanol instead of ethanol [23].

As cases surged in April 2021, cities like Phnom Penh were running out of hospital beds for COVID-19 cases. The government converted hotels and convention centers into dedicated COVID-19 treatment centers (Fig. 7). At first, all COVID-19 patients required to be hospitalized at government facilities, but the government later released guidelines for home treatment of patients with mild symptoms [24]. However, currently only a small number of patients are treated at home [25]. At the end of April 2021, private facilities were given permission to test and treat COVID-19, but only a few do so [26, 27].

**Fig. 7:** Hotels and convention centers are temporarily converted into dedicated COVID-19 treatment facilities

Against the backdrop of this widespread impact on the citizens of Cambodia, we conducted this review article to better understand the situation of healthcare workers in nephrology and dialysis patients and the challenge they face in providing and receiving essential medical care.

## The situation of healthcare providers in nephrology during the COVID-19 pandemic in Cambodia

To help us better understanding of the big pictures against our existing information, we have made a semi-structured telephone interviews with 7 colleagues healthcare providers in nephrology (5 doctors and 2 nurses) and 5 hemodialysis patients from 1 private and 3 public hemodialysis centers in Phnom Penh to find out about their situation during lockdown amid the COVID-19 pandemic in Cambodia. All interviewed doctors and nurses were continuing to work during the pandemic and lockdown. During the strict lockdown period, they initially found it extremely hard to travel across the city just to get to work because there were so many checkpoints along the way (Fig. 8). After arriving to work, these healthcare workers had more work than usual because of safety measures to prevent them being infected with the virus, such as wearing a surgical mask and face shield, limiting access to drinks, washing their hands more frequently, and performing simple infection control measures such as cleaning surfaces with alcohol or bleach according to the center’s policy. There was no increase in salary. Most centers do not have enough isolation spaces for hemodialysis sessions, so all patients are treated in a single space. Thus, the risk of one positive patient spreading the infection to the entire patient community is a major concern.

**Fig. 8:** Examples of traffic jams at checkpoints, April 17, 2021. Photo on the right: AFP

The healthcare providers also reported being victims of discrimination. A nurse told us that she was not allowed extend the lease for her rented room because the owner asked her to find another place to reside at request of nearby room renters. Other healthcare felt it was not safe to stay with their loved ones. They put themselves in isolation by staying on a separate floor, renting a place to stay, or staying at their workplace when possible.

Hemodialysis centers have been faced with a sharp increase in expenses for PPE, which is in limited supplies. At all the centers, revenue did not increase during these periods. Most centers required staff to at least wear surgical masks. Face shields and protective gowns were provided only by 1 center. Alcohol spray is routinely used for disinfection of beds and surfaces at all centers, and ultraviolet light disinfection is scheduled for use at 3 centers. For the safety of staffs and other patients, patients with fever or respiratory symptoms were asked to get a COVID-19 PCR test and wait for 2–3 days to receive the result before hemodialysis was allowed. Sometimes, patients returned with fluid retention or electrolyte imbalance as complications while waiting for or after receiving the PCR test result. Meanwhile, 1 center experienced a significant increase in the number of patients it treated, from roughly 300 patients in February to 400 cases in March, and about 450 cases in April. The reasons given for this increase were newly purchased hemodialysis machines in February, renovation to create more spaces, improvement of service, and most patients having difficulty traveling to other centers. None of the centers provides hemodialysis to patients with a diagnosis of COVID-19. COVID-19 patients who require hemodialysis are referred to a dedicated COVID-19 treatment facility. At only 1 of the 4 centers, 1 hemodialysis patient with COVID-19 was referred to a COVID-19 treatment facility, and no follow-up information could be obtained. Only 2 hemodialysis patients in 1 center have been vaccinated against COVID-19. No information about home hemodialysis or peritoneal dialysis was available.

Regarding vaccination of hemodialysis patients, there is a lack of medical information and guidelines that healthcare workers in nephrology can rely on in order to advise patients. Moreover, they are concerned about side effects of the vaccines and their safety profiles in hemodialysis patients. The healthcare workers were also concerned that if hemodialysis patients experience any health problem after vaccination, regardless of whether it is related to the vaccine, they will be blamed by the patient’s family for recommending the vaccination. Thus, doctors at hemodialysis centers said that they preferred not to discuss vaccination with patients or, if asked, told patients to wait and see.

## Challenges for hemodialysis patients during COVID-19 pandemic in Cambodia

Hemodialysis patients also experienced difficulties due to the pandemic and public health measures. Some patients had to eat salted dried fish or meat or canned food because of shortages of fresh food or difficulty in traveling.

During the COVID-19 pandemic and lockdown periods, access to healthcare has become even more difficult for hemodialysis patients. One reason for this was that these patients were being treated at centers far from their homes. Another reason was that most general medical clinics in Cambodia do not see patients who are on hemodialysis, even for simple complaints during normal times. In addition, patients with fever or respiratory symptoms were often turned away from one clinic after another.

Hemodialysis dosing was another challenge for the patients because of difficulty traveling during the initial strict lockdown period. Traffic jams at checkpoints and the number of the checkpoints were prominent barriers for all patients. At the beginning of the lockdown, traveling patients sometimes waited at checkpoints for up to 2 h due to the chaotic traffic conditions, with many people traveling in various directions getting stopped at the checkpoints.

The challenges would become even greater if a family member has COVID-19. Normally, many hemodialysis patients depend on family members to help with medical expenses and to take them to the hemodialysis center. Family members who have COVID-19 would regret not being able to provide this assistance, and the patients would have difficulty accessing the care they need.

For general safety during the pandemic, in-center hemodialysis rules have become stricter. Patients are required to wear a facemask and/or an optional face shield at some centers. Family members or escorts are no longer allowed to enter the unit with the patient, and patients are not allowed to eat inside the hemodialysis center.

Most of the hemodialysis patients we interviewed regarded end-stage kidney disease (ESKD) and the need for hemodialysis as end-of-life conditions and thus did not think it matters whether they are vaccinated against COVID-19. Also, some patients thought COVID-19 vaccines are not recommended for people with poor general health based on misinformation that spread via social media. They had also heard that hemodialysis and ESKD are conditions that cause poor immune status and that vaccines would not be safe for them.

## Opinion of the authors

Notwithstanding the well-intentioned attempts by the government to contain the spread of the virus, both the pandemic and the interventions made to contain it have a negative impact on society. People of all backgrounds, ethnicities, and income levels are under great pressure from COVID-19.

During the lockdown, healthcare workers in nephrology continued to work, but they had difficulty traveling to work, were prone to burnout, and had insufficient incentives. The layout of most hemodialysis centers is susceptible to the transmission of respiratory infections, so it was prudent that extra precautions were taken, including establishing stricter rules and not seeing patients with fever or respiratory symptoms until after a negative PCR test. However, measures steps placed constraints on healthcare workers in nephrology, who have been under considerable pressure, and added another layer of difficulties for the patients.

Because they have to frequently travel to receive treatment, hemodialysis patients have faced especially large socio-economic hardship while also being at especially high risk of SARS-CoV-2 infection. Moreover, they have a higher mortality rate compared with patients with many other conditions. When food access was limited, patients could not follow an appropriate hemodialysis diet and experienced complications such as fluid retention and electrolyte imbalance. For accessing hemodialysis care, travel restrictions both between provinces and within cities and the concentration of hemodialysis facilities in cities have together been a burden on top of ESKD during a time of economic hardship.

Vaccination is the solution. Vaccines have been shown to be safe and effective for hemodialysis patients and should be provided to them with high priority. It is unfortunate that misinformation about the vaccines has spread considering the extremely low risk of the vaccines compared with the very real risks of mortality and complications in hemodialysis patients. Authorities, as well as nephrology societies and their members, should speak with one voice as advocates for hemodialysis patients to remove of the many obstacles they face to encourage them to get vaccinated.

## Conclusion

Fortunately, there has not been a high incidence COVID-19 among hemodialysis patients in Cambodia, and the situation of the pandemic might improve in the coming months following the stringent measures and policies put in place by the Royal Government of Cambodia to contain the spread of the virus. Now, Cambodian nephrologists, nurses, dialysis technicians, allied health professionals, and ESKD patients are making their best efforts to fight against COVID-19. However, the burden on them is great. We hope for the swift and successful rollout of the vaccination program, which—as we are starting to see in countries around the world—can turn the tide of the COVID-19 pandemic.

## Data Availability

Data sharing is not applicable to this article as no datasets were generated or analyzed during the current study.

## Appendix

The content of this manuscript was presented in the NGO UBPI International Internet Dialysis-related COVID-19 Meeting among Cambodia, Vietnam, Mongolia, and Japan on May 15 and 16, 2021.

## Abbreviations

CKD: Chronic kidney disease
COVID-19: Coronavirus disease
ESKD: End-stage kidney disease
HD: Hemodialysis
JSDT: Japanese Society for Dialysis Therapy
MOH: Ministry of health
PCR: Polymerase chain reaction
PHEIC: Public Health Emergency of International Concern
PPE: Personal protective equipment
SARS-CoV-2: Severe acute respiratory syndrome coronavirus 2
UV: Ultraviolet
WHO: World Health Organization
